# Intermittent Hypoxia Effect on Osteoclastogenesis Stimulated by Neuroblastoma Cells

This article has been retracted.

**DOI:** 10.1371/journal.pone.0105555

**Published:** 2014-08-22

**Authors:** Vasantha Kumar Bhaskara, Indra Mohanam, Meena Gujrati, Sanjeeva Mohanam

**Affiliations:** 1 Department of Cancer Biology and pharmacology, University of Illinois College of Medicine, Peoria, Illinois, United States of America; 2 Department of Pathology, University of Illinois College of Medicine, Peoria, Illinois, United States of America; Faculté de médecine de Nantes, France

## Abstract

**Background:**

Neuroblastoma is the most common extracranial pediatric solid tumor. Intermittent hypoxia, which is characterized by cyclic periods of hypoxia and reoxygenation, has been shown to positively modulate tumor development and thereby induce tumor growth, angiogenic processes, and metastasis. Bone is one of the target organs of metastasis in advanced neuroblastoma Neuroblastoma cells produce osteoclast-activating factors that increase bone resorption by the osteoclasts. The present study focuses on how intermittent hypoxia preconditioned SH-SY5Y neuroblastoma cells modulate osteoclastogenesis in RAW 264.7 cells compared with neuroblastoma cells grown at normoxic conditions.

**Methods:**

We inhibited HIF-1α and HIF-2α in neuroblastoma SH-SY5Y cells by siRNA/shRNA approaches. Protein expression of HIF-1α, HIF-2α and MAPKs were investigated by western blotting. Expression of osteoclastogenic factors were determined by real-time RT-PCR. The influence of intermittent hypoxia and HIF-1α siRNA on migration of neuroblastoma cells and *in vitro* differentiation of RAW 264.7 cells were assessed. Intratibial injection was performed with SH-SY5Y stable luciferase-expressing cells and *in vivo* bioluminescence imaging was used in the analysis of tumor growth in bone.

**Results:**

Upregulation of mRNAs of osteoclastogenic factors VEGF and RANKL was observed in intermittent hypoxia-exposed neuroblastoma cells. Conditioned medium from the intermittent hypoxia-exposed neuroblastoma cells was found to enhance osteoclastogenesis, up-regulate the mRNAs of osteoclast marker genes including TRAP, CaSR and cathepsin K and induce the activation of ERK, JNK, and p38 in RAW 264.7 cells. Intermittent hypoxia-exposed neuroblastoma cells showed an increased migratory pattern compared with the parental cells. A significant increase of tumor volume was found in animals that received the intermittent hypoxia-exposed cells intratibially compared with parental cells.

**Conclusions:**

Intermittent hypoxic exposure enhanced capabilities of neuroblastoma cells in induction of osteoclast differentiation in RAW 264.7 cells. Increased migration and intratibial tumor growth was observed in intermittent hypoxia-exposed neuroblastoma cells compared with parental cells.

## Introduction

Neuroblastoma is the most common extracranial solid tumor in childhood [1], [2] and arises from embryonic neural crest tissue [2]–[4]. The most frequent sites of occurrence are the adrenal gland and the retroperitoneal region. Neuroblastoma is characterized by diverse clinical behaviors ranging from spontaneous regression to a highly aggressive disease, which is resistant to all currently available treatment modalities [5]. The majority of neuroblastoma patients present with metastatic dissemination at diagnosis and patients continue to have a poor prognosis despite intensive multimodality therapy [6], [7].

Hypoxia, a common feature of malignant tumors, contributes to the development of aggressive phenotype, resistance to radiation therapy [8] and chemotherapy, and is predictive of an overall poor outcome [9]–[15]. Furthermore, some studies have identified a relationship between tumor hypoxia and distant metastatic disease [16]–[18]. Intermittent hypoxia frequently arises in solid tumors as a result of improper neovascularization and irregular blood flow which is responsible for hypoxia and reoxygenation phases. The occurrence of intermittent hypoxic episodes varies significantly in rapidly growing malignant tumors [19]–[22].

Hypoxia can induce hypoxia inducible factor (HIF)-1α expression [23], which in turn increases the transcription of a number of downstream target genes involved in metabolism, proliferation, apoptosis, angiogenesis, and metastasis [15], [24], [25]. HIF proteins are composed of an α-subunit, HIF-1α, HIF-2α, or HIF-3α, and the constitutively present dimerization partner ARNT/HIF-1β. HIF-1α levels are controlled by regulated proteolysis through an oxygen-sensitive mechanism [24]. HIF-1α stabilization occurs more robustly as a result of intermittent hypoxia compared with chronic hypoxia [22], [26].

Bone is one of the preferential targets for metastatic neuroblastoma [27]. The presence of bone/bone marrow metastasis is associated with significant tumor aggressiveness and is responsible for an unfavorable prognosis despite high-dose chemotherapy and autologous hematopoietic stem-cell transplantation [28], [29]. To invade the bone, tumor cells produce factors that increase the osteoclast differentiation of hematopoietic precursor cells and the bone-resorbing activity of osteoclasts. This study was undertaken to investigate the effects of conditioned medium (CM) derived from intermittent hypoxia-exposed neuroblastoma cells on osteoclast differentiation using RAW264.7 cells. We demonstrated that HIF-1α is stabilized in intermittent hypoxia-exposed cells and that stabilized HIF-1α in neuroblastoma cells can induce osteoclastogenesis in RAW 264.7 cells.

## Materials and Methods

### Ethics statement

This study was performed in accordance with the guidelines and approval of the Institutional Animal Care and Use Committee of the University of Illinois, College of Medicine at Peoria, Peoria IL USA.

### Cell Culture

The human neuroblastoma SH-SY5Y cells and mouse monocyte/macrophage RAW 264.7 cells were obtained from the American Type Culture Collection (ATCC, Manassas, VA) and were cultured in DMEM supplemented with 10% fetal bone serum, penicillin(100 units/ml) and streptomycin (100 µg/ml) and maintained at 37°C in 5% CO_2_. Hypoxia was achieved by incubating cells in a humidified 5% CO_2_ atmosphere at 37°C in an incubator, in which the oxygen tension was held at 1%. To prepare CM, neuroblastoma cells were plated in 100-mm tissue culture dishes. Following overnight incubation, the medium was replaced with serum-free medium and cultured for 24 h. The supernatants were collected and filtered through a 0.22 µm syringe filter, aliquoted, and stored at −80°C until testing. The CM used in RAW 264.7 cells consisted of one-half volume neuroblastoma CM and one-half volume 2X RAW 264.7 cells growth medium.

### Establishment of intermittent hypoxia preconditioned cells

SH-SY5Y human neuroblastoma cells were exposed to 10 cycles of hypoxia and reoxygenation. Each cycle consisted of a period of 48 h in 1% hypoxia followed by 24 h recovery under normoxic conditions. During the reoxygenation period, the medium was changed. Afterwards, studies were performed using intermittent hypoxia-conditioned cells expressing increased levels of HIF-1α protein under normoxic condition unless otherwise stated.

### Plasmids

Pairs of complementary oligonucleotides against HIF-1α (sh-HIF-1α) and luciferase (sh-Luc) were synthesized, annealed and ligated into pGSH1-GFP according to the manufacturer's instructions (Genlantis San Diego, CA). Target sites in human HIF-1α and luciferase genes are as follows: HIF-1α, 5′- TTCAAGTTGGAATTGGTAG -3′ and luciferase, 5′- GATTATGTCCGGTTATGTA-3′. All inserted sequences were verified by DNA sequencing. Human HIF-1α cDNA (Origene) was cloned into the NotI site of pCI neo Mammalian Expression Vector (Promega).

### siRNA

Knockdown of HIF-1α or HIF-2α expression was achieved using HIF1α ON-TARGET plus SMART pool or HIF2α On-Target plus Smart Pool (Thermo-Dharmacon). ON TARGET plus Non-TARGET pool was used to control for non-specific effects.

### Transient and stable transfections

Parental cells or intermittent hypoxia-conditioned neuroblastoma cells were transfected under standard culture conditions with 40 ηM siRNA using the X-tremeGene (Roche) transfection reagent according to the manufacturer's instructions. For stable cell population selection, 24 h after transfection, parental cells were replated in growth medium with G418 (800 µg/ml). Colonies resistant to G418 were isolated and expanded. As a control, phCMV-Luc (Genlantis, San Diego, CA) expression vector was utilized to generate SH-SY5Y-Luc stable transfectants.

### Quantitative Real Time PCR (qPCR)

RNA was extracted from cultured cells using TRIzol reagent (Invitrogen) and reverse-transcribed using the Transcriptor First Strand cDNA synthesis kit (Roche) following the instructions of the manufacturer. RT-PCR was done using the iCycler (Bio-Rad) and IQ SYBR green Supermix (Bio-Rad). Relative expression values were obtained by the comparative ΔCT method normalizing CT-values to β-Actin or GAPDH. Primer sequences are provided in Table 1.

**Table 1:** List of primer sequences used for qPCR.

	Oligo Name	Sequence (5' to 3')
Human	HIF-1α F	TTCCAGTTACGTTCCTTCGATCA
	HIF-1α R	TTTGAGGACTTGCGCTTTCA
	HIF-2α F	GTGCTCCCACGGCCTGTA
	HIF-2α R	TTGTCACACCTATGGCATATCACA
	RANKL F	TGGATCACAGCACATCAGAGCAG
	RANKL R	ACTGGGGCTCAATCTATATCTCGAAC
	OPG F	GAAGGGCGCTACCTTGAGAT
	OPG R	GCAAACTGTATTTCGCTCTGG
	CXCR4 F	TCATCTACACAGTCAACCTCTACA
	CXCR4 R	GAACACAACCACCCACAAGTCATT
	VEGF F	AGGAGGAGGGCAGAATCATCA
	VEGF R	CTCGATTGGATGGCAGTAGCT
	β-Actin F	AGAAGGATTCCTATGTGGGCG
	β-Actin R	CATGTCGTCCCAGTTGGTGAC
Mouse	TRAP F	CACCCTGAGATTTGTGGCTGT
	TRAP R	CGGTTCTGGCGATCTCTTTG
	CaSR F	CGAGCACATCCCTTCAACCAT
	CaSR R	TAGTCGTCGTCGGCTGCAATT
	Cat K F	CCAGTGGGAGCTATGGAAGA
	Cat K R	CTCCAGGTTATGGGCAGAGA
	GAPDH F	CCCAGAACATCATCCCTGCAT
	GAPDH R	TCAGATCCACGACGGACACATT

### Western blot analysis

Cells were washed with PBS and lysed with lysis buffer (Cell Signaling Technologies). Equal amounts of protein were loaded onto SDS-PAGE gels, separated, and transferred onto nitrocellulose membranes. The membranes were blocked with 5% milk and incubated with the appropriate primary antibody. After washing, the membranes were treated with the corresponding horseradish peroxidase-conjugated secondary antibody. Blots were developed by using western lighting plus-ECL (PerkinElmer). Membranes were stripped and reprobed with β-actin antibody as a protein loading control.

### ELISA

Parental and intermittent hypoxia-exposed cells were transfected with non-targeted siRNA or siRNAs specific for HIF-1α or HIF-2α or treated with VEGF antibodies. After 36 h, cells were rinsed with PBS and serum-free DMEM was added. The CM was collected after 24 h. Concentrations of VEGF in the CM were determined by ELISA (R&D Systems) according to the manufacturer's instructions.

### Immunofluorescence

RAW 264.7 cells were exposed to growth medium with and without Receptor activator of nuclear factor-κB ligand (RANKL) or CM collected from parental or intermittent hypoxia-exposed neuroblastoma cells for 6 days. Medium was changed after 3 days. After 6 days, cells were fixed in methanol for 30 min at −20°C and then permeabilized with 0.3% Triton X-100 in PBS. After this, these cells were rinsed and blocked for one hour in 5% fetal bovine serum at room temperature. The cells were then incubated with anti- Ca2+-sensing receptor (CaSR) monoclonal antibody at 4°C overnight, after which cells were washed in PBS and then incubated with a secondary Alexa Fluor 488-conjugated anti-mouse antibody and 4',6-Diamidino-2-phenylindole (DAPI) for 1 h at room temperature. After extensive washing, imaging was performed using an Olympus fluorescent microscope.

### Monolayer wound migration assay

To perform migration assay, a scratch was made across the cell layer using a sterile pipette tip. The cells were washed twice with PBS and the medium was replaced. Cells were cultured to allow wound closure for 12 h, at which time pictures were taken with the Olympus microscope. Wound width was measured using a calibrated eyepiece graticule. The migration rate was calculated as the difference of the mean distance between both borderlines caused by scratching to the distance that remained cell-free after regrowing for 12 h.

### Osteoclast differentiation *in vitro*

RAW 264.7 cells were exposed to growth medium with and without rRANKL (100 ηg/mL) or CM collected from neuroblastoma cells. The cells were then allowed to grow for six days with the medium change after three days. Cells were stained for tartrate-resistant acid phosphatase (TRAP) by using the Leukocyte Acid Phosphatase Staining kit (Sigma-Aldrich) according to the instructions given in the kit. TRAP-positive multinucleated (three or more nuclei) cells were counted as osteoclasts in randomly selected fields under light microscope.

### TRAP activity

Cells were washed twice with PBS and solubilized in lysis buffer composed of 0.4 M sodium acetate pH 5.6 and 1% triton x-100. Samples were incubated with 10 mM p-nitrophenyl phosphate in 0.4 M sodium acetate buffer pH 5.6 containing 200 mM sodium tartrate. After 10 min of incubation, the reaction was terminated by the addition of 1 M NaOH. The absorbance of the samples at 410 nm was measured in an ELISA plate reader. Protein content in the lysates was measured by BCA reagent (Thermo Scientific, Rockford, IL, USA) and the results were expressed as ηmol/min/mg protein.

### Animal Experiments

The University of Illinois College of Medicine Peoria IL Animal Care and Use Committee (IACUC) approved the animal protocol used in this study. Luciferase-expressing neuroblastoma cells (5×10^5^ per mouse) were injected directly into the right tibia of anesthetized SCID mice using a Hamilton syringe equipped with a 29-gauge needle. Bioluminescence imaging was performed using Xenogen IVIS 200 small-animal imaging system as previously described [30]. Mice were sacrificed at day 35 post-implantation and tumor-injected tibias were harvested. Tibias were fixed overnight in 10% buffered formalin and decalcified for 3 weeks in 14% EDTA at pH 7.4 with changes every 48 to 72 h. Tissues were embedded in paraffin, and 5-µm thick sections were cut. Sections were stained for TRAP activity using reagent kits from Sigma-Aldrich to visualize osteoclasts.

### Statistical Analysis

The statistical significance of differences between data sets was determined using Student's t-test. P values of <0.05 were considered significant.

## Results

### Modulation of osteoclastogenic factors in human neuroblastoma cells upon intermittent hypoxia exposure

We examined the impact of intermittent hypoxia exposure on the expression of HIF-1α and HIF-2α in human neuroblastoma cells. Intermittent hypoxia-exposed cells were derived by exposing neuroblastoma SH-SY5Y cells to ten cycles of 48 h-hypoxic conditions followed by 24 h recovery under normoxic conditions. HIF-1α-siRNA and HIF-2α siRNA were used to knockdown HIF-1α and HIF-2α expression, respectively, in neuroblastoma SH-SY5Y cells. Real-time PCRs were done using primers specific to HIF-1α and HIF-2α. An increase in HIF-1α and HIF-2α mRNAs was observed in intermittent hypoxia-exposed cells compared with parental cells. Intermittent hypoxia-exposed cells treated with HIF-1α and HIF-2α-specific siRNA exhibited a decreased expression of HIF-1α and HIF-2α mRNAs, respectively, compared with intermittent hypoxia-conditioned cells exposed to non-targeted control (NTC) siRNA (Figure S1 A). The knockdown of HIF-1α and HIF-2α protein levels was confirmed by immunoblotting experiments using the HIF-1α and HIF-2α antibodies, respectively (Figure S1 B). An increase in mRNAs of HIF downstream genes VEGF and CXCR4 was observed in intermittent hypoxia-exposed cells compared with parental cells. Intermittent hypoxia-exposed cells treated with HIF-1α-specific siRNA exhibited a decreased expression of VEGF and CXCR4 mRNAs compared with intermittent hypoxia-exposed cells exposed to NTC siRNA (Figure S2).

To investigate the role of HIF-1α of neuroblastoma cells exposed to intermittent hypoxia in the regulation of osteoclastogenesis, mRNA levels of RANKL and osteoprotegerin (OPG) were quantitated by real-time RT-PCR. Intermittent hypoxia-exposure increased the abundance of RANKL expression in neuroblastoma cells. When HIF-1α expression was knocked-down with HIF-1α specific siRNA, the expression of RANKL was inhibited (Figure S3). OPG has been shown to inhibit RANK activation by competitively binding RANKL and was found to be decreased in intermittent hypoxia-exposed cells. Transfection of HIF-1α-siRNA in intermittent hypoxia-exposed cells resulted in the upregulation of OPG mRNA (Figure S3).

To examine the role of HIF-1α in induction of osteoclastogenic factors in neuroblastoma cells, we established neuroblastoma SH-SY5Y cells stably transfected with pCI-neo expression vector containing HIF-1α cDNA or pGSH1-GFP vector containing HIF-1α shRNA sequence or luciferase shRNA sequence. SDS PAGE analysis showed that HIF-1α stable transfectants expressed HIF-1α protein constitutively (Figure S4). HIF-1α protein was significantly reduced in HIF-1α knockdown cells exposed to hypoxia (1% O_2_, 24 h; Figure S4). mRNAs for VEGF, CXCR4, RANKL and OPG were analyzed in HIF-1α stable transfectants and HIF-1α knockdown cells. Relative expression levels of mRNAs for VEGF, CXCR4 and RANKL were significantly increased in HIF-1α transfectants and luciferase knockdown neuroblastoma cells exposed to hypoxia (1% O_2_, 24 h). A significant reduction in mRNAs for VEGF, CXCR4 and RANKL was observed in HIF-1α knockdown cells upon exposure to hypoxia (1% O_2_, 24 h; Figure S5). Decreased OPG mRNA was found in stable HIF-1α transfectants and the OPG mRNA increased in hypoxia exposed HIF-1α knockdown cells (Figure S5).

### Intermittent hypoxia exposure to neuroblastoma cells modulates *in vitro* osteoclastogenesis

To investigate the influence of intermittent hypoxia on neuroblastoma-induced osteoclastogenesis, CM from parental cells, intermittent hypoxia-exposed cells or stable transfectants of SHSY5Y cells (HIF-1α cDNA, luciferase shRNA or HIF-1α shRNA) were collected. The ability of these CM to induce osteoclast-like differentiation was determined using the TRAP assay. As shown in Figure 1A, RAW264.7 cells cultured in CM from intermittent hypoxia-exposed cells or HIF-1α transfectants had significantly higher TRAP activities than those cultured in the CM from parental cells. Cultures performed in the presence of CM derived from hypoxic HIF-1α knockdown cells displayed a lower number of osteoclastic cells than the cultures performed in the presence of CM of stable luciferase knockdown cells (Figure 1B). The collective data suggest that because of high levels of HIF-1α, intermittent hypoxia-exposed cells exhibit a higher ability to induce TRAP activity in RAW264.7 cells, thus facilitating osteoclast differentiation.

**Figure 1:** Effects of intermittent hypoxia exposure to neuroblastoma cells on *in vitro* osteoclastogenesis. RAW 264.7cells were supplemented with CM from the SH-SY5Y neuroblastoma cells and characterized for the osteoclastogenic response. (**A**) RAW 264.7cells were exposed to growth medium alone (control), growth medium with RANKL (100 ηg/ml) or CM from parental SH-SY5Y cells (N), intermittent hypoxia exposed (IH) cells, or stable transfectants (HIF-1α, shLuc and shHIF-1α) and were allowed to differentiate for six days under normoxic condition. The medium was changed after three days. CM from knockdown cells (shLuc and shHIF-1α) that were grown under hypoxia (1% O_2_, 24 h) were also evaluated. Cells were washed twice with PBS, fixed with 3.7% formaldehyde and stained for TRAP with Acid Phosphatase, Leukocyte (TRAP) kit according manufacturer's instructions. A representative image is shown. Arrow indicates cells multinucleated and TRAP-positive. (**B**) Multinucleated and TRAP-positive cells in each well were counted. Graphical representation of the number of osteoclast-like cells is shown. Values represent number of TRAP positive cells counted in ten different fields for each experiment from three independent experiments and expressed as mean ± SD. °°P<0.01 control versus RANKL; * P<0.05, **P<0.01 Parental (N) versus IH or HIF 1α; # P<0.05 shLuc/normoxia versus shLuc/hypoxia or shHIF 1α/hypoxia. (**C**) RAW 264.7cells were exposed to growth medium (control), growth medium with RANKL (100 ηg/ml) or CM from parental SH-SY5Y cells (N), IH cells, stable transfectants (HIF-1α, shLuc and shHIF-1α), or knockdown cells (shLuc and shHIF-1α) that were exposed to hypoxia (1% O_2_, 24 h) and were grown under normoxic condition for six days. The medium was changed after three days. Cells were assessed by real RT-PCR for the expression of TRAP, CaSR and Cath K mRNAs. Values are from three independent experiments in triplicates and expressed as mean ± SD. °°P<0.01 control versus RANKL; * P<0.05, **P<0.01 Parental (N) versus IH or HIF 1α; # P<0.05, ##P<0.01 shLuc/normoxia versus shLuc/hypoxia or shHIF 1α/hypoxia.

Furthermore, RAW 264.7 cells were exposed to growth medium with and without RANKL, CM from parental or intermittent hypoxia-exposed cells, or stable transfectants (HIF-1α cDNA, luciferase shRNA or HIF-1α shRNA) and were assessed by real RT-PCR for the expression of TRAP, CaSR and Cathepsin (Cath) K mRNAs. As the result show (Figure 1C), CM from intermittent hypoxia-exposed cells up-regulated the mRNA expression levels of TRAP, CaSR and Cath K in RAW 264.7 cells compared with the CM derived from parental cells. A significant increase in mRNAs for TRAP, CaSR and Cath K was observed in RAW 264.7 cells treated with CM from HIF-1α transfectants. CM of hypoxic HIF-1α knockdown cells caused a reduction in mRNAs for TRAP, CaSR and Cath K in RAW 264.7 cells (Figure 1C). Next, we evaluated CaSR protein levels by immunofluorescence and western blotting analysis. An increased expression of CaSR protein was observed in cells treated with CM from intermittent hypoxia-exposed cells compared with CM from parental cells (Figure 2A and 2B).

**Figure 2:** Effects of intermittent hypoxia exposure to neuroblastoma cells on CaSR expression in RAW 264.7 cells. (**A**) RAW 264.7 cells were exposed to growth medium (control), growth medium with RANKL or CM from parental SH-SY5Y cells (N), or intermittent hypoxia-exposed (IH) cells and cultured for six days under normoxia. The medium was changed after three days. Cells were fixed and labeled with CaSR antibodies and Alexa-594 antimouse-conjugated antibodies. Nuclei were stained with DAPI. RANKL-treated RAW cells served as a positive control for CaSR expression during osteoclastogenesis. A representative image is shown. Bar: 100 µm. (**B**) Cell lysates were analyzed for the levels of CaSR protein by Western blotting. The band intensity was measured and the protein level was normalized to the corresponding β-actin level. The results are expressed as relative quantity to the control (first lane of the blot).

### HIFs and VEGF on intermittent hypoxia-associated osteoclastogenesis *in vitro*

We examined the effects of intermittent hypoxia exposure on VEGF by measuring the amount of secreted VEGF protein in neuroblastoma cells. Intermittent hypoxia-exposed cells were transfected with NTC siRNA or HIF-1α-siRNA or HIF-2α-siRNA or HIF-1α + HIF-2α siRNAs (1∶1). Intermittent hypoxia-exposed cells secreted significantly increased VEGF protein compared with parental cells. Transfection of HIF-1α-siRNA or HIF-2α-siRNA or HIF-1α+HIF-2α siRNAs resulted in a marked decrease in the secretion of VEGF protein (Figure 3A).

**Figure 3:** Role of VEGF in intermittent hypoxia-exposed neuroblastoma cells-mediated osteoclastogenesis in RAW 264.7 cells. (**A**) Intermittent hypoxia-exposed (IH) neuroblastoma cells were transfected with NTC siRNA (siNTC), HIF-1α-siRNA (siHIF-1α), HIF-2α-siRNA (siHIF-2α) or HIF-1α siRNA+HIF-2α siRNA(1∶1 ratio) mix (siHIF-1α+siHIF-2α) and cultured under normoxia. After 36 h, the cells were washed and maintained in serum-free medium for 24 h.VEGF concentration in cell culture supernatants was determined by ELISA. Values are expressed as mean ± SD (n = 3). °°P<0.01 parental (N) versus IH; * P<0.05, **P<0.01 IH/siNTC versus IH/siHIF-1α or IH/siHIF-2α-siRNA or IH/siHIF-1α+siHIF-2α. (**B**) RAW 264.7 cells were exposed to growth medium (control), growth medium with RANKL, CM from parental SH-SY-5Y cells (N), IH cells or IH cells transfected with NTC siRNA (siNTC), HIF-1α-siRNA (siHIF-1α), HIF-2α-siRNA (siHIF-2α) or HIF-1α+HIF-2α siRNA (1∶1 ratio) mix (siHIF-1α+siHIF-2α) and were allowed to differentiate under normoxia. The medium was changed after three days. After six days, cells were washed twice with PBS, fixed with 3.7% formaldehyde and stained for TRAP. RANKL-treated RAW cells served as a positive control. TRAP-positive multinucleated cells containing three or more nuclei were counted under a light microscope. Values represent the number of TRAP positive cells counted in ten different fields for each experiment from three independent experiments and expressed as mean ± SD. °°P<0.01 control versus RANKL; **P<0.01 IH/siNTC versus IH/siHIF-1α or IH/siHIF-2α or IH/siHIF-1α+siHIF-2α. (**C**) IH cells were transfected with NTC siRNA (siNTC) or HIF-1α-siRNA (siHIF-1α) and CM were collected as described in Methods. Additionally parental, IH-siNTC, and IH-siHIF-1α cells were treated with VEGF antibodies and CM were collected. RAW 264.7 cells were exposed to growth medium (control), growth medium with RANKL, CM from parental or IH cells treated with NTC siRNA, HIF-1α-siRNA and/or VEGF antibodies and grown for six days with medium change after three days under normoxia. TRAP activity was assessed in cell lysates by the para-nitrophenyl phosphate hydrolysis assay. Results were normalized with total protein content of cultures and expressed as ηmol/min/mg protein. CM from RANKL-treated cultures served as a positive control. Values are expressed as mean ± SD (n = 4). °°P<0.01 control versus RANKL; **P<0.01 IH versus IH/VEGF Ab or IH/siHIF-1α.

We next examined the effects of HIFs knockdown on intermittent hypoxia-mediated osteoclastogenesis. CM of intermittent hypoxia-exposed cells enhanced osteoclastogenesis compared with control. On the other hand, CM from intermittent hypoxia-exposed cells transfected with HIF-1α-siRNA or HIF-2α-siRNA or HIF-1α + HIF-2α siRNAs significantly decreased the number of multinucleated TRAP positive cells, when compared with CM of intermittent hypoxia-exposed cells transfected with NTC siRNA (Figure 3B). Paralleling these data, RAW 264.7 cells exposed with CM from intermittent hypoxia-exposed cells treated with VEGF antibodies or HIF-1α siRNA exhibited a significantly reduced TRAP activity compared with CM of NTC siRNA- treated intermittent hypoxia-exposed cells (Figure 3C).

### Influence of intermittent hypoxia-exposed neuroblastoma cells on osteoclastogenic signaling pathways in RAW 264.7 cells

Earlier reports have indicated that the activation of MAPKs (ERK1/2, p38, JNK) play pivotal roles in stimulation of osteoclast differentiation [31], [32]. We examined the activation of MAPKs in RAW264.7 cells treated with CM from parental and intermittent hypoxia-exposed neuroblastoma cells by immunoblotting. Stimulation by RANKL (100 ηg/ml) markedly induced the phosphorylation of ERK, p38 and JNK in RAW264.7 cells (Figure 4A). However, no significant changes were observed in the levels of total MAPKs. As shown, CM from intermittent hypoxia-exposed cells markedly induced the activation of all three MAPKs in RAW 264.7 cells (Figure 4A).

**Figure 4:** Effects of intermittent hypoxia exposure to neuroblastoma cells on modulation of osteoclastogenic signaling pathways in RAW 264.7cells. (**A**) RAW 264.7 cells were exposed to growth medium (control), growth medium with RANKL (100 ηg/ml), CM from parental SH-SY5Y cells, or intermittent hypoxia-exposed (IH) cells. The cells were then allowed to grow for six days under normoxia with medium change after three days. The JNK, ERK and p38 activation states were determined by immunoblot analysis using antibodies specifically directed against the phosphorylated forms of the enzymes, compared to data obtained with antibodies directed against the unphosphorylated states of the kinases. (**B**) RAW 264.7 cells were exposed to CM from parental SH-SY5Y cells (N), IH cells or IH cells treated with 0.1 or 1 µM U0126 (MEK signaling pathway inhibitor), 2.5 or 5 µM SP600125 (JNK signaling pathway inhibitor) and 0.1 or 1 µM SB203580 (p38 signaling pathway) and cultured under normoxia. The medium was changed after three days. After six days, cultures were analyzed for TRAP-positive multinucleated cells containing three or more nuclei under a light microscope. A representative image is shown. (**C**) Graphical representation of the number of TRAP-positive multinucleated cells. Values represent the number of TRAP positive cells counted in ten different fields for each experiment from three independent experiments and expressed as mean ± SD. * P<0.05, **P<0.01 IH versus IH treated with SP600125 (2.5 or 5 µM) or SB203580 (0.1 or 1 µM).

Next, to determine which MAPK pathways are involved in intermittent hypoxia-exposed cells-induced osteoclastogenesis, the effects of specific MAPKs inhibitors, U0126 (MEK/ERK inhibitor), SB203580 (p38 MAPK inhibitor), and SP600125 (JNK inhibitor), were evaluated. RAW 264.7 cells were exposed to growth medium with and without RANKL (100 ηg/ml) or CM from parental, intermittent hypoxia-exposed cells or intermittent hypoxia-exposed cells treated with 0.1 or 1 µM U0126, 2.5 or 5 µM SP600125 or 0.1 or 1 µM SB203580. After six days, TRAP-positive multinucleated cells containing three or more nuclei were counted under a light microscope (Figure 4B). SP600125 andSB203580 revealed a very strong inhibitory effect on osteoclastogenesis in RAW 264.7 cultures supplemented with CM from intermittent hypoxia-exposed neuroblastoma cells while U0126 had no significant inhibitory effect (Figure 4C).

### Influence of intermittent hypoxia exposure on the migration of neuroblastoma cells

We next examined whether intermittent hypoxia-exposure affects tumor cell migration and whether changes in migration were due to altered HIFs expression. Wound-induced migration assay was performed using parental, intermittent hypoxia-exposed cells and intermittent hypoxia-exposed cells transfected with either HIF-1α-siRNA or HIF-2α siRNA or HIF-1α+HIF-2α siRNAs (Figure 5A). Intermittent hypoxia-exposed cells showed an increased migratory pattern compared with the parental cells. The mobility of intermittent hypoxia-exposed cells transfected with HIF-1α or HIF-2α specific siRNA was decreased in scrape wound migration assay compared with intermittent hypoxia-exposed cells transfected with NTC siRNA (Figure 5B).

**Figure 5:** Effects of intermittent hypoxia exposure on the migration of neuroblastoma cells. (**A**) Intermittent hypoxia-exposed (IH) cells were transfected with either NTC siRNA (siNTC), HIF-1α-siRNA (siHIF-1α), HIF-2α siRNA (siHIF-2α) or HIF-1α+HIF-2α siRNAs (1∶1 ratio) mix (siHIF-1α+siHIF-2α). Parental (N) and transfected cells were cultured at normoxia for 36 h, a scrape wound was made across the culture dish with a plastic pipette tip. The cells were washed twice with PBS and the medium was replaced. Cells were cultured to allow wound closure for 12 h, at which time pictures were taken with the Olympus microscope. Wound width was measured using a calibrated eyepiece graticule. A representative image is shown. (**B**) Graphical representation of monolayer wound-induced migration data. Values are expressed as mean ± SD (n = 4). °°P<0.01 Parental (N) versus IH; * P<0.05, **P<0.01 IH-siNTC versus IH-siHIF-1α or IH-siHIF-2α or IH-siHIF-1α+siHIF-2α.

### Intermittent hypoxia and osteolytic bone invasion of neuroblastoma tumors *in vivo*

To further validate the effects of intermittent hypoxia on osteoclastogenesis *in vivo*, we directly injected parental/Luc or intermittent hypoxia-exposed/Luc cells into the right tibia of 6-8-week-old female SCID mice. Tumor growth was imaged by bioluminescent imaging at five weeks after the implantation (Figure 6A). A significant increase of tumor volume was observed and reflected in the photon counts in animals that were injected with intermittent hypoxia-exposed cells compared with controls (Figure 6B). Next, we performed histologic examination of tumor tissues in bone. Consistently, TRAP staining revealed significantly higher osteoclasts at the bone/tumor interface from intermittent hypoxia-exposed cells-implanted animals compared with control animals (Figure 6C and 6D). These findings are consistent with the assessment that intermittent hypoxia plays a significant role in osteoclast differentiation *in vivo*.

**Figure 6:** Intratibial tumor growth. (**A**) Parental (N) and intermittent hypoxia-exposed (IH) cells (5×10^5^ in 25 µl PBS) stably expressing luciferase were directly injected into the right tibia of five to six week-old SCID mice. Bioluminescent activity was imaged in IVIS-100 system at 35 day after the implantation and photon counts were collected to reflect live tumor volume. (**B**) Quantification of bioluminescence **p<0.01, parental (N) versus IH cells. (**C**) Tibias were harvested, decalcified, sectioned, and stained for TRAP. A representative image is shown and the arrow indicates TRAP-positive osteoclasts. (**D**) Graphical representation of number of osteoclast-like cells, counted by microscopy after TRAP staining.**p<0.01, parental (N) versus IH cells.

## Discussion

Neuroblastoma is the most common extracranial solid tumor in childhood and is remarkable for its broad spectrum of clinical behaviors, including spontaneous regression or aggressive progression. Recent studies have shown that hypoxia can be an indicator of poor outcome for malignant neuroblastoma [33], [34]. It is well known that neuroblastoma cells exposed to intermittent hypoxia, which is characterized by cyclic periods of hypoxia and reoxygenation, undergo a complex cascade of changes [35]. Intermittent hypoxia has been shown to render tumors more invasive in animal models [36], [37] and enhance angiogenic processes and radioresistance in the vascular endothelium of tumors [21].

We found that intermittent hypoxia exposures increased the levels of HIF-1α and HIF-2α proteins and enhanced stem-like properties of neuroblastoma cells [35]. The expression of mRNAs of HIF downstream genes VEGF and CXCR4 was found to be increased in intermittent hypoxia-exposed cells. Further, HIF-1α siRNA significantly inhibited the VEGF and CXCR4 mRNAs in intermittent hypoxia-exposed cells. Our results are in line with other studies which have shown that HIF-1α and HIF-2α subunits contribute to VEGF transcriptional activation in hypoxic neuroblastoma cells [38]. It has been found that CXCR4 overexpression was associated with increased incidence of metastasis *in vivo* in a xenograft model as well as correlating with the pattern of metastatic spread in neuroblastoma patients [39], [40]. Our results show that neuroblastoma cells exposed to intermittent hypoxia exhibit increased levels of mRNAs associated with angiogenesis and metastasis by stabilizing HIFs (HIF-1α and HIF-2α).

Tumor cells produce factors that stimulate osteoclastic bone resorption [41], [42]. In the present study, we examined whether intermittent hypoxia treatment contributed to the development of bone metastases by measuring the mRNAs of osteoclastogenic factors in intermittent hypoxia-exposed cells. Osteoclast differentiation factor RANKL is the prime dominator of the differentiation pathway of precursor cells to osteoclasts and is also responsible for the activation of osteoclasts [43], [44]. In addition, OPG is a decoy receptor for RANKL that regulates the functional state of RANKL [41]. A putative HIF-1α binding element resides at the RANKL promoter region [45] and induced HIF-1α was found to be associated with an increase in RANKL mRNA expression in intermittent hypoxia-exposed neuroblastoma cells. Earlier studies have shown that OPG expression level was down-regulated in hypoxic human oral squamous carcinoma cells and HIF-1α knock-down significantly increased OPG expression under hypoxic condition [46]. Our studies also demonstrated that intermittent hypoxia represses OPG expression in human neuroblastoma cells in part via HIF-1α induction.

Because HIF-1 α is a “master regulator” of many adaptive responses to hypoxia [47], we investigated the effects of HIF- α forced expression and HIF- α knockdown under hypoxia on the expression of osteoclastogenic factors. We transfected neuroblastoma cells with a plasmid encoding sh-HIF-1α sequence or HIF-1α cDNA. HIF-1α overexpression significantly increased the expression of osteoclastogenic factors in neuroblastoma cells under normoxic conditions whereas knockdown of HIF-1α abrogated the intermittent hypoxia -mediated increased expression of osteoclastogenic factors.

The RAW 264.7 mouse monocytic cell line was chosen as a source of preosteoclast cells in our *in vitro* model since the RAW 264.7 cell line has been shown to readily differentiate into osteoclasts upon exposure to recombinant RANKL [48], [49]. Since neuroblastoma frequently metastasizes to bone and causes osteolysis in bone metastases [27], [50], we examined the effects of CM of intermittent hypoxia-exposed cells on the differentiation of RAW 264.7 cells. In our study, intermittent hypoxia treatment increased osteoclast formation induced by neuroblastoma cells, as demonstrated by the strong induction of the formation of TRAP positive cells. We also studied the effects of CM of stable HIF-1α transfectants and CM of hypoxic stable HIF-1α knockdown cells on osteoclastogenesis *in vitro*. Our findings clearly show that increased HIF-1α levels induced the formation of active osteoclasts, as assessed from the numbers of TRAP-positive multi-nucleated cells. Previous studies have shown that HIF-1α expression promoted the progression of bone metastases in breast cancer [51], [52].

Osteoclast differentiation is associated with the up-regulation of specific genes in response to RANKL. Osteoclasts contain abundant TRAP and are responsible for bone resorption.

In this study, well known marker genes of osteoclasts, such as TRAP, Cath K and CaSR were greatly up-regulated in RAW 264.7 cells treated with CM of intermittent hypoxia-exposed cells. Cath K is abundantly and predominantly expressed in osteoclasts where it is localized in the lysosomes, in the ruffled border and in the resorption lacunae on the bone surface [53]. Mentaverri et al [54] have shown that the CasR exerts a direct effect on osteoclastogenesis using bone marrow cells isolated from CaSR−/− mice as well as dominant negative CaSR-transfected RAW 264.7 cells. The role of HIF-1α in induction of marker genes of osteoclasts was also studied using CM of stable HIF-1α transfectants and CM of hypoxic stable HIF-1α knockdown cells. Our findings clearly show that intermittent hypoxia enhances the osteoclastogenesis potential of neuroblastoma cells, in part, by HIF-1α stabilization.

Several studies have shown that VEGF enhances osteoclastogenesis [55]–[60]. In our studies, exposure to intermittent hypoxia significantly increased VEGF secretion, whereas treatment with HIF-1α-siRNA, HIF-2α-siRNA or HIF-1α+HIF-2α siRNAs resulted in a marked decrease in the secretion of VEGF protein. CM from intermittent hypoxia-exposed cells treated with siRNAs for (HIF-1α or HIF-2α or HIF-1α+HIF-2α) produced a significant decrease in TRAP-positive multi-nucleated cells in comparison with CM of NTC siRNA-treated intermittent hypoxia-exposed cells. This finding is consistent with previous studies showing that the hypoxic CM from human osteosarcoma cells treated with HIF-1α + HIF-2α siRNAs produced a significant decrease in TRAP-positive multi-nucleated cells and TRAP activity [60]. In our studies, CM of intermittent hypoxia-exposed cells induced TRAP activity which was inhibited by co-incubation with a neutralizing anti-VEGF antibody. These results suggest that intermittent hypoxia could influence osteoclastogenesis via secretion of VEGF under the control of HIFs.

MAPKs such as JNK, ERK and p38, have been reported to be activated by RANKL stimulation and to be associated with osteoclastogenesis [32], [61]. We have investigated how these signaling pathways are modulated in the process of intermittent hypoxia-exposed cell-mediated osteoclastogenesis. In our present observation, using RAW 264.7 cells, we found that CM from intermittent hypoxia-exposed cells significantly enhanced phosphorylation of JNK, ERK and p38. In addition, JNK inhibitor, SP600125, and p38 MAPK inhibitor, SB203580 strongly inhibited osteoclastogenesis in RAW 264.7 cells induced by CM from intermittent hypoxia-exposed cells. However, the ERK inhibitor, U0126, had no inhibitory effect on osteoclastogenesis enhanced by CM of intermittent hypoxia-exposed cells. These results demonstrated that intermittent hypoxia promotes osteoclastogenesis by activating p38 and JNK signaling pathways.

Cell migration is a critical step and a precondition for tumor invasion. In our studies, knockdown of HIF-1α or HIF-2α blocked the intermittent hypoxia-mediated increased migration pattern. It is well known that up-regulation of osteoclastogenesis is a necessary prerequisite for the ability of cancer cells to successfully colonize in osteolytic bone metastasis [62], [63]. Increased expression of osteoclastogenesis-associated genes in neuroblastoma cells can exacerbate their metastatic potential. Furthermore, osteoclastogenic factors secreted by neuroblastoma cells may propel a cascade of events that trigger osteoclastogenesis and elevated resorptive activity in the bone microenvironment. The progression of neuroblastoma bone metastases requires the establishment of functional interactions between neuroblastoma cells and bone cells. It has been shown that neuroblastoma cells injected directly into the femur of immunodeficient mice are capable of proliferating and stimulating osteolytic reaction of mouse bone [64]. In order to confirm the role of intermittent hypoxia in neuroblastoma bone metastasis, parental and intermittent hypoxia-exposed neuroblastoma cells were inoculated into the bone of SCID mice by intratibial injection. Our results suggested that intermittent hypoxia exposure in neuroblastoma cells increased osteolytic neuroblastoma tumor establishment and growth in the bone environment.

## Conclusions

In summary, the results of our study indicated that intermittent hypoxia exposures promoted expression of osteoclast differentiation associated genes in neuroblastoma cells. CM from intermittent hypoxia-exposed cells markedly induced the activation of JNK, ERK and p38 signaling pathways in RAW264.7 cells. Intermittent hypoxia enhanced neuroblastoma cells survival and growth in tibias, and thereby contributed to the progression of bone metastasis (Figure 7).

**Figure 7:** Schematic representation of the role of intermittent hypoxia in enhancement of neuroblastoma-mediated osteoclastogenesis.

## Supporting Information

Figure S1 **Expression of HIF-1α and HIF-2α expression in intermittent hypoxia-exposed neuroblastoma cells.** (**A**). Intermittent hypoxia-exposed (IH) cells were transfected with either NTC siRNA (siNTC), HIF-1α-siRNA (siHIF-1α), HIF-2α siRNA (siHIF-2α) or HIF-1α/HIF-2α siRNA (1∶1 ratio) mix (siHIF-1α+ siHIF-2α). Parental and transfected cells were cultured for 36 h at normoxia. Total RNA was extracted using Trizol and cDNA was generated by reverse transcription. Real-time PCRs were done using primers specific to HIF-1α and HIF-2α. Values are expressed as mean ± SD (n = 4). °°P<0.01 Parental (N) versus IH; **P<0.01 siNTC versus siHIF-1α or siHIF-2α. (**B**) Parental (N) and IH cells were transfected with and without siRNAs targeting HIF-1α and/or HIF-2α, cultured for 36 h at normoxia, lysed with RIPA buffer containing protease inhibitors. Cell extracts were subjected to electrophoretic analysis through SDS-PAGE. The knockdown of HIF-1α and HIF-2α was confirmed by immunoblotting using the HIF-1α and HIF-2α antibodies respectively. The band intensity was measured and each protein level was normalized to the corresponding β-actin level. The results are expressed as relative quantity to the parental (N) cells (first lane of each blot).
(TIF)

Figure S2 **Effect of intermittent hypoxia exposure on the expression of hypoxia-inducible genes in neuroblastoma cells.** Parental (N) and intermittent hypoxia-exposed (IH) cells were transfected with either NTC siRNA (siNTC) or HIF-1α-siRNA (siHIF-1α) and cultured under normoxia for 36 h. Total RNA was extracted using Trizol and cDNA was generated by reverse transcription. Real-time PCRs were done using primers specific to VEGF and CXCR4. Values are expressed as mean ± SD (n = 4). °°P<0.01 parental (N) versus IH cells; **P<0.01 siNTC versus siHIF -1α.
(TIF)

Figure S3 **Effect of intermittent hypoxia preconditioning on the expression of osteoclastogenic factors in neuroblastoma cells.** Intermittent hypoxia-exposed (IH) cells were then treated with either NTC siRNA (siNTC) or HIF-1α siRNA (siHIF-1α) under normoxic condition for 36 h. mRNAs for RANKL and OPG were quantified in parental (N) and IH cells treated with siRNAs using iCycler IQ. Values are expressed as mean ± SD (n = 3). °°P<0.01 IH versus normoxia; * P<0.05: **P<0.01 IH-siNTC versus IH-siHIF 1α.
(TIF)

Figure S4 **Expression of HIF-1α in HIF-1α stable knockdown and overexpression transfectants.** SH-SY5Y cells were transfected with pCI-neo expression vector containing HIF-1α cDNA, pGSH1-GFP vector containing HIF-1α shRNA sequence or luciferase shRNA sequence, and stable transfectants were generated. Stable HIF-1α shRNA and luciferase shRNA transfectants were also subjected to hypoxia (1% O_2_, 24 h)). Parental and transfectants were lysed with RIPA buffer containing protease inhibitors and cell extracts were subjected to electrophoretic analysis through SDS-PAGE. The overexpression and knockdown of HIF-1α in stable transfectants was confirmed by immunoblotting using the HIF-1α antibodies. The band intensity was measured and each protein level was normalized to the corresponding β-actin level. The results are expressed as relative quantity to the parental (N) cells (first lane of the blot).
(TIF)

Figure S5 **Expression of osteoclastogenic factors in HIF-1α overexpression and knockdown cells.** HIF-1α stable transfectants (HIF-1α), HIF-1α knockdown (shHIF-1α) and luciferase knockdown (shLuc) cells were generated in SH-SY5Y cells as described in Methods. mRNAs for VEGF, CXCR4, RANKL and OPG were quantified using iCycler IQ in parental cells (control) and in stable transfectants grown at normoxia (HIF-1α, shHIF-1α and shLuc) or stable transfectants exposed to hypoxia (shHIF-1α and shLuc; 1% O_2_, 24 h). Values are expressed as mean ± SD (n = 3). Intermittent hypoxic exposure enhanced neuroblastoma cells capabilities in induction of osteoclast differentiation in RAW 264.7 cells °P<0.05, °°P<0.01 control versus HIF 1α; * P<0.05,**P<0.01 shLuc-normoxia versus shLuc-hypoxia; # P<0.05, ##P<0.01 shLuc-hypoxia versus shHIF-1α-hypoxia.
(TIF)
